# Computer Security Issues and Legal System Based on Cloud Computing

**DOI:** 10.1155/2022/8112212

**Published:** 2022-07-11

**Authors:** Hui Li

**Affiliations:** School of Marxism, Xi'an Fanyi University, Xi'an710105, Shaanxi, China

## Abstract

To effectively improve the security and accuracy of computer information storage, a computer security problem and legal system based on cloud computing are proposed. Firstly, this article details the evolution of cloud computing, its characteristics, architecture, and application status of cloud computing in detail. Second, we discussed security strategies to ensure the confidentiality and integrity of cloud computing information, focuses on the data encryption technology of cloud data security, and designs and implements the data backup and recovery system based on the cloud platform. The core layers of the system are the system layer and data operation layer. The system uses multithreading technology based on epoll and thread pool to improve the efficiency of data transmission. At the same time, the basic visual page is realized, and users can use the page to create a convenient operating system. Finally, the system is built in the laboratory environment and tested as a whole. The test results show that through the performance comparison with the current commonly used systems, it is found that the system in this paper has a certain improvement in data transmission rate, but the utilization rate of node CPU is as high as 40%, which leads to certain requirements for node CPU performance. Therefore, the system meets the functional requirements proposed in the design. Compared to the existing system, its performance has been found to meet the actual requirements of use, proving that the system is accessible and efficient.

## 1. Introduction

With the rapid development of computer science and technology, computer network information technology is also developing day by day, and the penetration of computer network technology in all walks of life is becoming more and more extensive. Under this background, cloud computing technology came into being. Cloud computing is a large data processing technology that processes and shares data by combining computer technology and network technology. The use of cloud computing in computer applications can provide users with a large number of network resources. Computer users can obtain cloud resources anytime and anywhere through computing technology so that each computer user can enjoy the massive information resources and data information in the network [1]. The main manifestations of the new age of science and technology are cloud computing, big data technology, and artificial intelligence. Cloud computing technology has been involved in many fields such as social finance, urban transportation, education, and medical treatment [2]. With the continuous improvement of society's dependence on computer technology, the problem of network security is becoming more and more obvious. In order to ensure the security of computers in the context of cloud computing, we must establish a perfect network security supervision and management mechanism, build a perfect network security legal guarantee system, and widely carry out network legislation throughout the country. However, there are still prominent problems in today's network security legal governance [3, 4].

Computer security mainly includes the security of computer stored data and computer hardware safety [5]. The data in the computer is the core resource of the whole computer. The essence of various operations performed by the computer is to make effective use of the data. It can use resources in different places at the same time and organically integrate edge resources [6]. Now, more and more people begin to use cloud computing, and various applications based on cloud platforms emerge in endlessly. Baidu cloud disk, 360 cloud disk, and other applications are becoming more and more popular, which also confirms this situation [7]. However, because the application data in the cloud platform are stored in the server, in this case, if the system data is lost or damaged, it will have a disastrous impact on a large number of users [8]. Therefore, how to ensure that the cloud platform can realize high-capacity data-efficient backup and timely data recovery in case of disaster has become a subject that must be considered. At present, it seems that the use of data backup and recovery systems to back up system data can restore data in a timely manner in the event of system failures and data loss, effectively improve information security, reduce losses, and ensure reliable operation of system [9]. The paper proposes a new data backup and recovery system under a cloud platform for specific laboratory projects and environments. Through the master-slave backup of management nodes and data nodes, the reliability of the system itself is effectively guaranteed. Through the backup and recovery of system data, the data security of the system is greatly improved [10].  Figure 1 shows a study of computer security issues and countermeasures in cloud computing.

## 2. Literature Review

Data is the core of the current information society, which is very important for all walks of life. Therefore, how to ensure data security has become a key issue for people to consider, and data backup technology also came into being. Early data backup is mainly cold backup through a tape drive, optical disc, and disk. When there is a devastating failure in the computer room, these backups also stored in the computer room cannot play an effective backup role at all. Rehman et al. [11] play an important role in protecting network information in a cloud computing environment in order to effectively improve the security and availability of data and realize the improvement and creation of storage system, so as to give priority to hot data access to corresponding levels, and improve reading and writing efficiency [11]. Dastres and Soori [12] believe that the connection and storage of traditional storage technologies are realized through the data interface with the host. In the process of small demand for data storage, they use the storage mode to connect with each other, and there are problems in the process of creating the connection. The main server side will affect the operation of data. In the process of increasing storage, the server carrying capacity is constantly improving, reducing the operation efficiency [12]. Geetha et al. [13] proposed that the computer network security virtual filtering system based on cloud computing can map the development trend of the market. Users can connect with each other in the mobile terminal and data center and calculate according to their own needs [13]. Durakovskiy et al. [14] believe that a network storage system is mainly applied to network technology, and realizes the hardware design of storing a large amount of data information by separating data information from the server [14]. Kumar et al. [15] proposed that the network security virtual filtering system based on cloud computing technology creates the management domain and virtual machine domain through the host computer. The virtual domain is the calling interface of the upper virtualization layer to operate the system in the virtual software platform [15]. Airesurquiza et al. [16] believe that cloud computing is an Internet-based computing method. In this way, shared software and hardware resources and information can be provided to computers and other devices on demand. The needs of a large number of users can be met [16, 17]. Tan et al. [17] use virtualization mode to improve processing efficiency. Users can use cloud computing through the network, and each request is distributed to multiple servers [18]. Dhulavvagol et al. [19] proposed that the computer network security virtual filtering system based on cloud computing can map the development trend of the market. Users can connect with each other in the mobile terminal and data center and calculate according to their own needs [19].

Based on this research, this paper proposes a computer security problem and legal system based on the background of cloud computing, designs the overall performance and function of the system according to the conditions used by the cloud platform, and gives the overall framework of the system. It mainly carries out modular design for the core level of the system, system level, and data operation level. The data operation layer is divided into modules such as data synchronization, data backup, data recovery, and concurrent transmission. In the data synchronization module, the master-slave node data synchronization is realized through the snapshot transmission of the master node. In the data backup module, three backup types are supported as follows: full backup, incremental backup, and differential backup. In the data recovery module, appropriate backup data is selected to improve the recovery efficiency. Finally, the system is built in the laboratory environment and tested as a whole.

## 3. Research Methods

### 3.1. Cloud Computing Technology

#### 3.1.1. Cloud Computing Classification

As modern society continues to evolve, humanity is entering an era of information explosion. With the increasing number of application users, the increasing demand for computing power, and the increasing security requirements, enterprises have to increase investment in hardware equipment to meet the growing needs. At the same time, the requirements for system operation and maintenance are increasing day by day to ensure the safety and reliability of hardware [20]. More importantly, this growth model is carried out in the form of an index. Therefore, cloud computing technology with simple use, low cost, and easy access to resources has gradually come to people's attention.

The service modes of cloud computing are divided into the following three categories:

1. Infrastructure is a service. Users purchase servers, storage, and other hardware equipment from cloud service providers, which save their own space on the physical level and can be used whenever hardware needs to be used.
2. Platform is a service. Instead of providing hardware equipment to users, cloud service providers provide services to users in the form of middleware [21, 22]. Users do not need to care about the type of hardware equipment they use but can directly carry out their own development on the provided platform.
3. Software is a service. For such services, users do not need to carry out any other operations on the services provided; they can use them directly, and they do not need to care about the underlying platform and infrastructure. These layers are shielded from users in software as a service. This type of service is mainly aimed at the direction of mobile Internet. For software application development on mobile devices such as mobile phones, when using the back-end as a service method, the server side of the application is provided by the cloud service provider, which helps mobile application developers get rid of the background development problems and focus on the development of mobile desktop applications, which helps to speed up the development process and save development funds [23, 24].

#### 3.1.2. Cloud Computing Features

Cloud computing has five basic features:

1. Self-service on demand. Users can add or delete resources applied to cloud service providers by analyzing their own needs.
2. Extensive network access. Users can access the cloud through various types of terminals, not just personal computers.
3. Resource sharing. It provides services to users in a unified form by integrating different resources in space. Users do not need to care about where they use resources.
4. Fast elasticity. The speed of providing or releasing resources is very fast. For users, the available resources they see are almost unlimited. Users can purchase and use resources at will without considering the total amount of remaining resources.
5. Services are measurable. The cloud system can make rational use of the resources of the whole system independently. At the same time, the whole process can be clearly and reliably provided to service providers and service users through a visual interface by means of detection software.

### 3.2. Computer Data Security

#### 3.2.1. Classification of Data Backup

Computer data backup is the process of copying the entire or part of a data set in a system to another memory in a certain way to prevent data loss due to human factors, such as operating errors or system failures. Data backup can be classified according to different angles. Based on common backup strategies, data backup can be divided into three types as follows: full backup, incremental backup, and differential backup [25].

1. Full backup. Full backup refers to backing up all the data in the system to the specified storage. When the system needs to be restored in case of failure, full backup can restore the system at one time. However, corresponding to its convenient recovery, full backup requires a lot of time and system resources. If full backup is carried out every time, a large amount of redundant data will be generated, resulting in a great waste of storage space and increasing the storage cost of users.
2. Incremental backup. Incremental backup, as the name suggests, means that each backup is based on the part added by the previous data. This backup method has high efficiency and occupies few system resources due to few backup data. The disadvantage is that each incremental backup needs to be performed in the order of backup in order to restore the system to the state at the time of final backup. If an incremental backup is lost, the recovery of the whole system will be affected.
3. Differential backup. The time required for backup is also in between. When the system fails to recover, it only needs two backups: full backup and differential backup. The performance of recovery is also better.

#### 3.2.2. Data Recovery Technology

Data recovery technology is mainly divided into two types. One type is called disaster recovery technology. This mainly refers to the way that the system can still recover quickly through previous data backup after system failure or disaster through various backup methods introduced before, so as to ensure that the system can recover normal services as soon as possible. The use scenario of this method usually requires existing data backup. Using the previous data backup can quickly and accurately restore the system to the network. This disaster recovery technology is also the main recovery technology used in this system. Another narrow sense of data recovery technology refers to the technology that fails to recover data directly through backup after data damage or loss, but needs to recover data through lower technical means. According to different recovery objects, this technology can be divided into software recovery technology for operating system and file system recovery; hardware recovery technology for hard disk track and disk chip recovery [26, 27].

For the general recovery process, disaster recovery technology is usually used for data recovery when there is data backup and the data backup can be used normally. In case of data backup loss or data backup hardware damage, software or hardware recovery technology shall be used for data recovery according to different conditions. Therefore, in the context of cloud computing, build a set of network security legislation systems that can serve the broadest masses of the people, so that the public can more comprehensively and scientifically realize the importance of relevant laws and regulations for the construction of network security environment, and win the recognition of the broadest masses of the people for network security legislation and regulations.

### 3.3. Analysis and Design of Computer Data Backup and Recovery System Based on Cloud Computing

#### 3.3.1. Overall System Structure Design

The system uses a layer design that includes five basic layers as follows: the user layer, the system layer, the application layer, the data operation layer, and the storage layer. The general structure diagram of the system is shown in Figure 2. The marked system layer and data operation layer are the core design levels of this paper.

#### 3.3.2. System Layer Management Node Module Design

As one of the main functional layers of the system in this article, the system layer is responsible for managing the entire system, such as registering the system log and passing user instructions to the appropriate modules, including recording the system log, transmitting user instructions to appropriate modules, realizing load balancing to optimize the load, confirming the user identity, and judging whether the operation of system nodes has faults [28]. The core of the system layer is the management node. Therefore, in this section, the function of the management node is modularized to meet the overall needs of the system. Since the management node realizes many functions, only several main modules are given here, as shown in Figure 3.

#### 3.3.3. Modular Design of Data Operation Layer

The key functions such as data backup and recovery are realized in this layer. Since this layer mainly carries out data transmission, data security should be considered first. For the data operation layer, there are two main methods to improve security.

1. Encrypt data during transmission to ensure the safety of data during transmission. Symmetric encryption. The encryption key and decryption key of this method are the same, so its encryption and decryption speed is fast, but its security has been tested. In the process of secret key transmission, if it is stolen, the thief can easily decrypt the ciphertext data. At the same time, because each communication object will save a secret key, a large number of secret keys will be generated when there are too many objects, which is not conducive to secret key management. Asymmetric encryption. The encryption key and decryption key of this method are different, which are generally called the public key and private key. However, the public key is generally long and takes a lot of time to complete the encryption process. Therefore, in the actual use process, the user's private key encryption and public key decryption are often used to realize the asymmetric encryption process. One-way encryption. This method is also called hash encryption. It is mainly an encryption method that encrypts data through a hash algorithm to generate short and fixed-length eigenvalues. Because the characteristic values generated by each file through one-way encryption are different, and when the file data changes, the characteristic values of the new file are also different from those of the original file. Therefore, this method is mainly used to detect whether the data is completely transmitted during transmission, and judge whether the transmitted data has been modified.
2. Data integrity inspection. Data transmission is not a stable process, and the data after transmission may be missing due to network reasons or hacker damage. Therefore, before and after data transmission, the sum of transmission data calculation and verification is needed. The source end verification and destination verification sum are compared to determine whether the data completed by transmission is missing. At present, hash algorithms such as MD 5 are commonly used to test data integrity. MD 5 (message digest Algorithm 5), algorithm is a widely used hash algorithm. The main idea is to group the data with 512 bits and continue to divide each 512-bit group into 16 32 bit subpackets. After that, these subpackets are transformed into four 32 bit packets by the algorithm. Finally, the four packets are cascaded, and the generated 128-bit hash value is then obtained eigenvalue. The modular division of the data operation layer is shown in Figure 4. In this modular division, only the core modules are listed. Next, this paper will design these modules.

### 3.4. Cloud Data Security Based on Homomorphic Data Encryption

#### 3.4.1. Complete Homomorphic Encryption Algorithm

Homomorphic encryption algorithms include four main algorithms: key generation algorithm, data encryption algorithm, data decryption algorithm, and appropriate evaluation algorithm. This paper will use the symmetric homomorphism encryption algorithm created by Craig gentry. The algorithm designed in this paper is as follows:

*(1) Encryption algorithm*. The encrypted variables are *p*, *Q*, and *R*. the variable p is positive and odd, and *Q* stores a large integer. *P* and *Q* are assigned when generating the key. *P* belongs to the encrypted key, and the variable *r* stores a random number during encryption. For plaintext *m*, we calculate

(1) $$\begin{array}{c} c=m+2r+pq. \end{array}$$

The ciphertext can be obtained.

*(2) Decryption algorithm*. For plaintext

(2) $$\begin{array}{c} \text{m}=\left(c\mathrm{mod}p\right)\mathrm{mod}2. \end{array}$$

Since *pq* is much greater than 2*r* + *m*, there are

(3) $$\begin{array}{c} \left(c\mathrm{mod}p\right)\mathrm{mod}2=\left(m+2r\right)\mathrm{mod}2=m. \end{array}$$

#### 3.4.2. Proof of Homomorphism of Algorithm

For example, the existing plaintext *m*_1_ and *m*_2_ are grouped, and then the encrypted ciphertext can be obtained by encrypting the two groups as follows:

(4) $$\begin{array}{c} c_{1}=m_{1}+2r_{1}+pq_{1},\\ c_{2}=m_{2}+2r_{2}+pq_{2}. \end{array}$$

For plaintext,

(5) $$\begin{array}{c} m_{3}=m_{1}=m_{2}. \end{array}$$

Because

(6) $$\begin{array}{c} c_{3}=c_{1}+c_{2}=\left(m_{1}+m_{2}\right)=2\left(r_{1}+r_{2}\right)+p\left(q_{1}+{}_{q}^{2}\right). \end{array}$$

As long as (*m*_1_+*m*_2_)=2(*r*_1_+*r*_2_) is far less than *P*, there are

(7) $$\begin{array}{c} c_{3}=\left(c_{1}+c_{2}\right)\mathrm{mod}p=\left(m_{1}+m_{2}\right)+2\left(r_{1}+r_{2}\right). \end{array}$$

Through the above proof, algorithm can realize the addition operation in homomorphism.

The method encrypts the data in the process of transmission, which can prevent data loss or embezzlement. Only through the key can the data be encrypted and restored. However, only users have the key, which increases the security of cloud computing for data. Because the fully homomorphic encryption algorithm is adopted, cloud computing can perform various operations and processes on the data but cannot obtain the plaintext in the data. This method can save time in the process of data encryption and transmission. Only users can decrypt the data, but the cloud is responsible for other data processing, which improves the processing efficiency and ensures the security and privacy of the data.

## 4. Result Discussion

### 4.1. Test Environment Construction

This system is a test platform built based on the laboratory environment. The system includes 2 terminals and 9 servers, which are connected through the switch. One of the two terminals is used as an administrator user and the other as an ordinary user. The 9 servers are divided into three categories: 2 servers are used as management nodes, including 1 master management node and 1 slave management node; five are used as data nodes, including one master data node, three slave data nodes, and one backup data node, and the remaining two are used as application servers. For the specific test environment, see Figure 5.

For the configuration details of each terminal and server, see Table 1.

### 4.2. Performance Test

Compare this system with the commonly used data backup and recovery system and analyze the advantages and disadvantages of this system and other systems.

#### 4.2.1. Test and Analysis of Factors Affecting System Performance

Since the system backup performance is related to many factors, the following tests are conducted for several parameters affecting the system in this paper.

*(1) Single File Size has an Impact on System Backup Performance*. Test the data with the same total amount of data and different file sizes. After multiple tests, take the average value as the final result and generate a histogram, as shown in Figure 6.

When a single file increases, because the system divides the file by size during backup transmission and realizes the function of multiple nodes acquiring data for transmission at the same time, when the file increases, the number of nodes that can transmit the file at the same time also increases, and the backup efficiency will increase. A large number of server connection operations are often required for the transmission of small files, which will also lead to the decline of the system transmission rate.

The total amount of backup data has an impact on the system backup performance. Backup data of different sizes, compare the average running rate, and take the test average as the final result after multiple tests. The histogram is shown in Figure 7.

As the total amount of backup information increases, the system transfer rate increases until it stabilizes. The reason for this is that when the amount of data transmitted by the system is small, creating and releasing thread pool resources (Figure 8) will occupy a large system overhead. However, with the increase in the total number of files, the thread pool model can improve the data transmission efficiency of the system until the transmission rate tends to be stable.

#### 4.2.2. System Performance Comparison Test and Analysis

Next, the system performance is tested. The main focus of the test is the rate of data recovery and backup, and the utilization of system resources in the recovery process. It can be seen from the above that the commonly used data backup and recovery systems in the market include the beitejia backup system and data protector system (hereinafter referred to as DP system). The test method is to select backup data of a specified size for backup and recovery. The main focus is on the rate of data recovery and backup, as well as the utilization of system resources in the recovery process. It can be seen from the above that the commonly used data backup and recovery systems in the market include the beitejia backup system and data protector system (DP system for short). Next, the above two systems are compared with the system in this paper to verify the performance of the system in this paper.

(1) Data Backup Test: use different sizes of backup data to test, and compare the backup duration, compare the backup time, CPU, and memory usage of the three systems with the same amount of data. The results of the data backup efficiency are shown in figure 8. As you can see from the results, the system mentioned in this article is slightly better than the other two systems in terms of data transfer speed. The main reason is that the thread pool design based on epoll multiplexing has been realized, which has significantly improved the data transmission efficiency.

Figure 9 shows the comparison of the average CPU utilization during data backup of the three systems. Because the system uses a thread pool to transmit data, it occupies more CPU resources. DP system has obvious advantages in CPU occupancy.

Figure 10 shows the comparison of the average memory utilization rate during data backup (Figure 11) of the three systems. The memory utilization rates of the three systems are basically the same.

(2) The data recovery test also uses different sizes of recovered data to test and compares the recovery time, CPU, and memory occupancy of the three systems under the same amount of data. The average recovery rate of the system is shown in Figure 11. The system in this paper is still slightly better than the other two systems.

Figures 12 and 13 show the comparison of average CPU utilization and memory during data recovery of the three systems. In terms of CPU utilization, the DP system is still better, and the memory utilization of the three systems is still basically similar.

From the above test results, it can be seen that the system in this document meets the basic functional requirements of the system for backing up and recovering data on the cloud platform, and the system reliability is high. Comparing the performance of the systems currently in use, the system described in this article has improved the data transfer rate to some extent, but found that the relatively high speed of the node CPU usage makes certain demands on the system. Through the analysis of the test results, it shows the feasibility of the system in practical application.

### 4.3. Legal System Construction to Solve Computer Security Problems in the Context of Cloud Computing

#### 4.3.1. Strengthening Legislation on Cyber Security Issues

In the context of cloud computing, the Legislative Division for Strengthening Computer Network Security will establish a “Cyber Security Personal Data Protection Law” to integrate best practices in the protection of personal data in similar countries and regions, and establish a personal information security system. The relationship between users' personal information and their private lives is getting closer. Compared to laws and regulations, special legal protection regulations can have a real legal effect. The legislative process should define the scope of personal information, protect the confidentiality of personal information, crack down on violations, and impose fines to standardize the legal regulation of the personal information of network users. In addition, as e-commerce technology develops, issues such as transaction information disclosure and platform price fraud are becoming more acute, and relevant e-commerce protection laws need to be enacted to effectively regulate the e-commerce market. Effectively protect the legitimate interests of users based on the new level of the media, make clear regulations, increase controls, manage and punish such illegal actions, and severely punish such behavior, thus ensuring a harmonious and orderly network security for network users.

#### 4.3.2. Refinement of Legal Provisions on Network Security Issues

The Law on Cyber Security contains strategic provisions such as network sovereignty, protection of the network operating environment, protection of network products, network services, and information security, and provides relevant legal and regulatory guarantees for network security. The detailed terminology is relatively broad, and some details and specific regulations need to be further implemented and refined, as well as relevant regulations. Therefore, the relevant departments should improve and create the relevant legislation, update and improve the relevant laws in a timely manner based on the actual development of the network information, and fill the gaps in the monitoring and management of the implementation of the network legislation. For example, due to the nonstandard legislation of the real-name system on the Internet, some network users do not have real-name system restrictions in their network operations, and network security issues cannot be effectively addressed. In response to this problem, on the one hand, network users must create the knowledge to disable network information. When a host leaves a website, criminals must cancel their information to prevent the reuse of network name information. The technology is constantly being improved in order to provide stronger legal, regulatory, and policy support for the development of network security in the context of cloud computing, the perfect development of network security, and the reduction of network security issues in the cloud application.

## 5. Conclusion

As a popular technology, cloud computing has more and more applications based on the cloud platform. If data on the cloud platform is damaged or lost, it will lead to serious consequences. Therefore, in order to ensure the effective development of the network security environment system and support the improvement of the legal governance system, the relevant departments should support the further development of legislation in this area based on the basic concept of cloud computing. Network society under the cloud computing background actively introduces excellent and advanced laws and regulations. The data backup and recovery system designed and implemented in this paper provide users with a more reliable cloud platform data protection scheme. The system is built in the laboratory environment, and the overall test of the system is carried out. Through the test results, the indexes of the system are analyzed. The results show that the system meets the functional requirements of the model. Compared to the existing system, its performance has been found to meet real needs, which confirms the system's accessibility.

## Figures and Tables

**Figure 1:** Research on computer security issues and countermeasures in cloud computing.

**Figure 2:** Overall system architecture.

**Figure 3:** Module division of management node.

**Figure 4:** Module diagram of data operation layer.

**Figure 5:** Schematic diagrams of the test environment.

**Figure 6:** Test of influence of data block size on the transmission rate.

**Figure 7:** Impact test of total data on the transmission rate.

**Figure 8:** Comparison of average data backup rates of three systems.

**Figure 9:** Comparison of average CPU utilization during data backup of three systems.

**Figure 10:** Comparison of average memory utilization during data backup of three systems.

**Figure 11:** Comparison of average data recovery rates of three systems.

**Figure 12:** Comparison of average CPU utilization during data recovery of three systems.

**Figure 13:** Comparison of average memory utilization during data recovery of three systems.

**Table 1:** Test machine configuration list.

Machine type	Number of machines	Operating system	IP allocation
PC terminal	2	Windows 7	Administrator: 191.167.1.40 Ordinary users: 191.167.1.41
Management node	2	Debian 8.0	Main node: 191.167.1.101 Slave node: 191.167.1.102
Data node	5	Debian 8.0	Main node: 191.167.1.103 Slave node: 191.167.1.104-6 Management node: 191.167.1.107
Application node	2	Debian 8.0	Node 1: 191.167.1.108 Node 2: 191.167.1.109

## Data Availability

No data were used to support this study.
